The article "Medical Image Classification Algorithm Based on Visual Attention Mechanism-MCNN" was published in 2021. Journal: Oxid Med Cell Longev.

# Medical Image Classification Algorithm Based on Visual Attention Mechanism-MCNN

**DOI:** 10.1155/2021/6280690

**Published:** 2021-02-19

**Authors:** Fengping An, Xiaowei Li, Xingmin Ma

**Affiliations:** ^1^School of Physics and Electronic Electrical Engineering, Huaiyin Normal University, Huaian 223300, China; ^2^System Second Department, North China Institute of Computing Technology, Beijing 100083, China

## Abstract

Due to the complexity of medical images, traditional medical image classification methods have been unable to meet the actual application needs. In recent years, the rapid development of deep learning theory has provided a technical approach for solving medical image classification. However, deep learning has the following problems in the application of medical image classification. First, it is impossible to construct a deep learning model with excellent performance according to the characteristics of medical images. Second, the current deep learning network structure and training strategies are less adaptable to medical images. Therefore, this paper first introduces the visual attention mechanism into the deep learning model so that the information can be extracted more effectively according to the problem of medical images, and the reasoning is realized at a finer granularity. It can increase the interpretability of the model. Additionally, to solve the problem of matching the deep learning network structure and training strategy to medical images, this paper will construct a novel multiscale convolutional neural network model that can automatically extract high-level discriminative appearance features from the original image, and the loss function uses the Mahalanobis distance optimization model to obtain a better training strategy, which can improve the robust performance of the network model. The medical image classification task is completed by the above method. Based on the above ideas, this paper proposes a medical classification algorithm based on a visual attention mechanism-multiscale convolutional neural network. The lung nodules and breast cancer images were classified by the method in this paper. The experimental results show that the accuracy of medical image classification in this paper is not only higher than that of traditional machine learning methods but also improved compared with other deep learning methods, and the method has good stability and robustness.

## 1. Introduction

Medical imaging is a technique and process for noninvasively obtaining a part of a tissue image of a human body. Differences in the clinical experience of doctors may result in a decline in the quality of medical image analysis and may even lead to misdiagnosis and missed diagnosis of patients [1, 2]. A reliable computer-aided diagnostic system can improve the above situation. Therefore, improving the performance of medical imaging film computer-aided diagnosis systems has become an important issue that has attracted the attention of relevant scholars [1]. Image classification technology can carry out preliminary analysis and understanding of medical images and can effectively identify the corresponding lesion areas, thus, assisting doctors in pathological diagnosis [2, 3]. Although there are many current image classification methods, they can be generally divided into image classification methods based on traditional machine learning and image classification methods based on deep learning [4–6].

Medical image classification methods based on traditional machine learning mainly include linear discriminant analysis, artificial neural networks, support vector machines, *k*-nearest neighbor classifiers, and genetic algorithms. Lee et al. [7] used a combination of genetic algorithms and linear discriminant methods to classify 62 malignant nodules and 63 benign nodules. They achieved certain effects, but the generality of the model was weak. Suzuki et al. designed a large-scale training artificial neural network for the diagnosis of benign and malignant reduction in false positives and pulmonary nodules in nodule detection [8, 9] and achieved a good recognition effect. However, the adaptive ability was poor. Way et al. [10] used a support vector machine to classify benign and malignant lung nodules by extracting the two-dimensional texture. However, it was less effective in classifying smaller lung nodules. Firmino et al. [11] used support vector machine algorithms to train 420 lung cancer cases and then classified smaller lung nodules. The classification accuracy rate was 94.4%. However, it is still not ideal for the benign and malignant recognition of small lung nodules. Yu et al. [12] classified squamous cell carcinoma and adenocarcinoma in nonsmall cell lung cancer by automatic microscopic pathological image features. It had a classification effect on lung adenocarcinoma and lung squamous cell carcinoma of more than 70%. However, it did not have a good solution for classification between large cell carcinoma and squamous cell carcinoma and adenocarcinoma in lung cancer. Through the above analysis, it can be seen that although such methods have been promoted and applied to a certain extent in medical image classification, certain effects have been achieved. However, they cannot be adaptively matched to medical image characteristics. They cannot extract the medical feature information contained in the image, which makes the overall classification effect of these methods less than ideal. There is a certain gap between the classification effect and the requirements for assisting doctors in performing effective diagnoses [13, 14].

In 2006, Hinton and Salakhutdinov first proposed the concept of deep learning in the first issue of Science magazine [15], which introduced feature learning. The emergence of deep learning technology provides a new idea and technical approach for solving the problems existing in traditional machine learning medical image classification methods. Deep learning technology [15] has been widely used in computer vision [16–18], speech recognition [19, 20], and video analysis [21–23]. Therefore, research on medical image classification based on deep learning has attracted extensive attention and in-depth research by scholars in the industry. Anthimopoulos et al. [24] used a deep learning network to classify an adult chest radiograph database and achieved good results. Plis et al. [25] and Suk et al. [26, 27] used a deep belief network and a self-encoder to classify brain magnetic resonance imaging, which can be used to determine if a patient has Alzheimer's disease. Zhang et al. [28] used a restricted Boltzmann machine (RBM) to automatically extract image features from shear waveform elastography and used this method to classify breast tumors. The classification accuracy rate reached 93.4%. Cheng et al. [29] used a stacked autoencoder to classify breast ultrasound lesions and nonnodules. The classification performance was 10% higher than the general method. Kawahara and Hamarneh [30] used a multibranch CNN to classify skin lesions, which achieved a certain classification effect. Esteva et al. [31] trained CNN using a dataset of 129,450 clinical images. The CNN also classified and recognized cell carcinoma and benign seborrheic keratosis. The experimental results showed that the classification level of skin cancer by CNN reached the level of a dermatologist. Bidart et al. [32] developed a method for autolocalization of breast cancer tissue sections using a fully convolutional neural network and divided the nuclear images from breast cancer tissue sections into lymphocytes, benign epithelial cells, and malignant epithelial cells. The final classification accuracy rate was 94.6%. Setio et al. [33] input the 9 differently oriented patches extracted from the candidate images into separate networks and combined them in the fully connected layer to obtain the final classification output. The experimental results were more obvious than the general methods. Nie et al. [34] analyzed the nature of MRI by training 3DCNN to assess the survival rate of patients with high glioma. Payan and Montana [35] and Hosseini-Asl et al. [36] used 3D convolutional neural networks to classify patients with Alzheimer's disease. The accuracy and robustness of the classifier were superior to several conventional classifiers. Through the above analysis, deep learning theory has been widely promoted and applied in the field of medical image classification. It has also achieved good results. However, since medical images have more distinct and different feature information than natural images, the self-characteristics of medical images must be fully considered when constructing a deep learning model. Therefore, a deep learning model can obtain better medical image classification effects, which is one of the most difficult problems in building a deep learning model. Additionally, due to the current deep learning network structure and training strategies, medical images are less adaptable. This finding points to the accuracy of medical image classification based on deep learning. To fully exploit the characteristics of medical images, first, by introducing a visual attention mechanism, it is possible to locate and extract effective information for medical images. Second, reasoning can be achieved at a finer granularity by introducing a visual attention mechanism. Finally, the attention mechanism increases the explanatory form of the model by visualizing attention. Additionally, to solve the problem of matching the deep learning network structure and training strategy to medical images, this paper constructs a novel multiscale convolutional neural network model that can automatically extract high-level discriminative appearance features from the original image, and the loss function uses the Mahalanobis distance optimization model to obtain a better training strategy, which can improve the robust performance of the deep learning network model. The medical image classification task is completed by the above method. Based on this, this paper proposes a medical classification algorithm based on a visual attention mechanism-multiscale convolutional neural network.

Section 2 of this paper explains the deep learning model based on the visual attention mechanism proposed in this paper.  Section 3 systematically describes the multiscale convolutional neural network model proposed in this paper.  Section 4 introduces a medical classification algorithm based on a visual attention mechanism-multiscale convolutional neural network.  Section 5 analyzes the medical image classification algorithm proposed in this paper and compares it with the mainstream medical image classification algorithm. Finally, the full text is summarized and discussed.

## 2. Deep Learning Model Based on a Visual Attention Mechanism

### 2.1. Multiwheel Attention Memory Network Encoder

Given an image *f*, its category is *c*, denoted as *f*_*c*_ in this article. First, input the image into the standard long short-term memory network (LSTM) [37] and then use the long-short-term memory model to calculate the vector of the image as *V*_*f*_*c*__ ∈ *R*^*d*^. The specific calculation formula is

(1) $$\begin{array}{c} V_{f_{c}}={\text{LSTM}}^{f}\left(f_{c}\right). \end{array}$$

In the formula, all problems share the encoder LSTM^*f*^.

This paper proposes a network structure with multiple rounds of attention mechanisms, which is used to extract enough useful information from the cross-modal medical category fact memory and visual fact memory. It, thus, enables more accurate class identification *f*_*c*_.

The vector representation *V*_*fc*_ for the class identification problem *f*_*c*_ and the two memory banks *M*^*I*^ and *M*^*H*^ are associated therewith. The problem *V*_*fc*_ is first projected into the historical medical category memory *M*^*H*^ by the following formula to retrieve the category facts associated with the category identification question *f*_*c*_:

(2) $$\begin{array}{c} u_{0}=V_{f_{c}}, \end{array}$$

(3) $$\begin{array}{c} s_{i}=u_{j-1}\cdot m_{i}^{H},j=1,\cdots ,r., \end{array}$$

(4) $$\begin{array}{c} u_{j-1}=u_{j-1}+\overset{c-1}{\underset{i=0}{\sum }}\alpha_{i}m_{i},\alpha_{i}=\exp\left(s_{i}\right)/\overset{c-1}{\underset{i=0}{\sum }}\exp\left(s_{i}\right), \end{array}$$

where *r* represents the attention mechanism round. *s*_*i*_ is a measure of similarity between *u*_*j*−1_ and *m*_*i*_^*H*^. The result *u*_*j*−1_ is calculated each time through the projection problem to the category memory. This method treats the result as the latest expression of the problem *f*_*c*_ carrying the category. The neural network is then used to continue projecting it into the visual fact memory to retrieve the computationally related visual category facts. The specific formula is as follows:

(5) $$\begin{array}{c} h=\tanh\left(W_{f,h}M^{I}⊕\left(W_{u}u_{j-1}+b_{h}\right)\right), \end{array}$$

(6) $$\begin{array}{c} p^{I}=\text{soft}\max\left(W_{p}h+b_{p}\right), \end{array}$$

(7) $$\begin{array}{c} u_{j}=u_{j-1}+\overset{196}{\underset{i=0}{\sum }}p_{i}^{I}m_{i}^{I}, \end{array}$$

where *W*_*i*,*h*_, *W*_*u*_ ∈ *R*^*k*×*d*^, and *b*_*h*_ ∈ *R*^*k*^. ⊕ marks the addition between the matrix and the vector. *h* is the output of the single-layer neural network obtained by the previous result obtained by the nonlinear hyperbolic tangent function. *W*_*p*_ ∈ *R*^*k*×*d*^ and *p*^*I*^ ∈ *R*^196^ represent the projection probability value (i.e., correlation) between each picture region and *u*_*j*−1_. The output *u*_*j*_ is obtained by projecting the visual memory. It also contains the category and visual fact information related to question *f*_*c*_. To date, the model has performed a single-round projection process for cross-modal memories. Then, the model proceeds to the next round of the cross-modal attention mechanism through equation (7) until the preset total round limit *r* is reached, which can solve the problem of information transfer and reasoning.

Alternate projection calculations for the category and visual fact memory through the *r*-round obtain *u*_*r*_ containing factual information that can answer question *f*_*c*_. Then, input it to the single-layer neural network to obtain the final output of the encoder, specifically

(8) $$\begin{array}{c} e_{c}=\tanh\left(W_{e}u_{r}+b_{e}\right), \end{array}$$

where *W*_*e*_ and *b*_*e*_ are the weights and offsets of the fully connected neural network, respectively. *e*_*c*_ is the final encoded output of the problem *f*_*c*_.

### 2.2. Generating and Discriminating Decoders

#### 2.2.1. Generating Decoder

Given the problem *f*_*c*_ and the encoder's final coded representation *e*_*c*_, its corresponding class *a*_*c*_ is generated by:

(9) $$\begin{array}{c} h_{0}=e_{c}, \end{array}$$

(10) $$\begin{array}{c} h_{i}={\text{LSTM}}^{g}\left(h_{i-1},x_{i-1}\right),i=1,\cdots ,\left|a_{c}\right|, \end{array}$$

(11) $$\begin{array}{c} p_{i}=\text{soft}\max\left(W^{g}h_{i}+b^{g}\right), \end{array}$$

where LSTM^*g*^ is a productive LSTM decoding network. *h*_*i*_ is the output of the *i*th training of LSTM^*g*^. *x*_*i*_ is the vector representation corresponding to the *i*-th category of the image *a*_*c*_. The length of *a*_*c*_ is ∣*a*_*c*_∣. *p*_*i*_ is the probability distribution of the category. During the training process, the method maximizes the probability of generating the correct category *a*_*c*_. In the test evaluation phase, the probability size of each candidate category is calculated first. All candidate categories are then ordered by probability in descending order.

#### 2.2.2. Discriminant Decoder

First, each candidate class is encoded by the following LSTM, which can obtain the corresponding vector expression:

(12) $$\begin{array}{c} h_{a_{i}}={\text{LSTM}}^{d}\left(a_{i}\right),i=1,\cdots ,N, \end{array}$$

where LSTM^*d*^ is the encoder for all candidate categories and shares weights. *h*_*a*_*i*__ is the final encoded output of the *i*th candidate category *a*_*i*_. Then, the degree of similarity *s*_*i*_ between the vectors is calculated by the point multiplication similarity:

(13) $$\begin{array}{c} s_{i}=e_{c}\cdot h_{a_{i}}. \end{array}$$

Then, all the similarities {*s*_1_, *s*_2_, ⋯, *s*_*N*_} obtained are spliced together and input into a softmax classifier, which then calculates the posterior probability of all candidate categories; namely,

(14) $$\begin{array}{c} p_{a}=\text{soft}\max\left(s_{1}\Theta s_{2}\Theta \cdots s_{N}\right), \end{array}$$

where Θ represents the stitching operation, and *p*_*a*_ is the probability distribution for the candidate category. In the training process, the method maximizes the discriminant probability of the correct category *a*_*c*_. In the verification and testing phase, it can sort it from large to small directly by the posterior probability of each candidate category.

## 3. Multiscale Convolutional Neural Networks

### 3.1. Network Structure

The multiscale convolutional neural network model proposed in this paper consists of the following three parts: input data processing, feature extraction of deep learning models, and similarity calculation of different features. Its overall structure is shown in Figure 1. Since deep learning technology has a strong generalization ability in learning high-level visual features, this paper introduces deep convolutional neural network into the model and uses it as an automatic feature extractor. Due to the particularity of medical images, the deep learning model proposed in this article contains a spatial pyramid pool. It is mainly used to extract rich and effective multiscale visual cues from different scale spaces of images and can extract fixed-dimensional feature vectors from medical images of different sizes/scales. Based on this, this paper proposes a multiscale convolutional neural network architecture, that is, a triple network architecture (three branch networks share parameters) and an improved triple loss function. First, it reorganizes the training samples into a large number of triples. In turn, it expands the size of the training set. Then, it uses deep convolutional neural networks to classify medical images.

The model first generates a large number of triple samples from the training set, which is then fed into a subnet shared by three parameters. The improved triplet loss function is used to force the distance between the similar image and the sample to be smaller than the dissimilar image pair. Additionally, the additional pairwise constraints push similar samples close to each other, reducing the intraclass variance. Given a training set {*Y*}, it can generate a large number of triplet images as input. The *i*-th triple is represented by *x*_*i*_ = (*y*_*i*_, *y*_*i*_^+^, *y*_*i*_^−^), where *y*_*i*_ represents a medical image with classification, *y*_*i*_^+^ represents another image of the same medical image, and *y*_*i*_^−^ represents medical images from different categories. The triple image (*y*_*i*_, *y*_*i*_^+^, *y*_*i*_^−^) is mapped from the image space to the specific feature space by three deep networks sharing the same parameter (*W*). The depth features extracted by the deep learning network are expressed as (*f*_*w*_(*y*_*i*_), *f*_*w*_(*y*_*i*_^+^), *f*_*w*_(*y*_*i*_^−^)), and then the similarity between any two images *y*_*i*_ and *y*_*j*_ is calculated according to their Mahalanobis distance, specifically

(15) $$\begin{array}{c} \begin{array}{c} D_{M}\left(y_{i},y_{j}\right)={\left(f_{w}\left(y_{i}\right)-f_{w}\left(y_{j}\right)\right)}^{T},\\ M\left(f_{w}\left(y_{i}\right)-f_{w}\left(y_{j}\right)\right), \end{array} \end{array}$$

where *M* is a semipositive definite matrix. The goal of the model is to learn an appropriate metric matrix from the feature space through an improved triple loss function, which can pull features of the same category of medical images closer together and push features belonging to different medical category images away from each other. This paper connects the improved triple loss function to the top of the deep network. After training the model, it can simultaneously obtain discriminative features and appropriate distance metric matrices to distinguish different categories of medical images.

### 3.2. Deep Convolutional Neural Network Model

The network layer in the multiscale triple convolutional neural network proposed in this paper is based on the ResNet-50 model and is composed of two layers. The filter size indicates the size of the convolution kernel and the number of channels. The output dimension represents height × width. The layer types of different network layers include convolution, block, residual module, maxpooling, SPP (space pyramid pooling layer), FC (full connection layer), and L2 (norm normalization layer).

The initial convolutional layer in the network contains 128 7 × 7 convolution kernels. Its step size is set to 1 × 1, and the initial maximum pooling layer size is 2 × 2. It is used to extract low-level local features and reduce the size of feature maps. Each residual module includes a plurality of residual functional layers, each of which consists of a stack of 3 consecutive convolutional layers. The convolution kernels of the three convolutional layers are 1 × 1, 3 × 3, and 1 × 1. The 1 × 1 convolutional layer is responsible for reducing the feature dimension so that the size of the 3 × 3 convolutional layer input and output is relatively small. The step size of the convolutional layer in each residual module is 1 × 1, except that the stride of Conv3_1 and Conv4_1 is set to 2 × 2, and the stride of Conv5_1 is set to 2 × 1. Deeper convolutional neural networks are difficult to optimize. Therefore, the shortcut connection mechanism in the residual module (multiple residual function layers) is applied to the deep neural network model [38], which can improve the depth of the deep network and obtain a more accurate recognition accuracy.

The spatial pyramid pooling layer can generate a fixed number of spatial windows whose size is proportional to the image size. In the network model of this paper, four different types of spatial windows are used: 1 × 1, 2 × 2, 4 × 4, and 8 × 8. They are used in the spatial pyramid pooling layer. This layer pools the response of each filter according to different spatial window types. The output of the spatial pyramid pooling layer is a fixed 2,048 M dimension vector, where *M* represents the total number of bins, and 2,048 is the dimension of the conv5_y layer. The resulting fixed-length feature is fed into the loss function via a fully connected layer. The spatial pyramid pooling layer can extract multilevel spatial pyramid pooling operations for feature maps to extract more discriminative multiscale appearance information. After passing through four residual modules and a spatial pyramid pooling layer, the network model is connected to a fully connected (800-dimensional) layer that determines the dimensions of the medical category feature vector. The final layer of the deep convolutional network model is an L2 normalization layer. It is used to normalize the medical image category features of the output of the fully connected layer. Each convolutional layer in the network is connected to a rectified linear unit (ReLU) (as an activation function) layer.

### 3.3. Loss Function and Optimization

Let *Y* = {*y*_*i*_^*p*^ | *i* = 1, 2, ⋯, *N*} denote a training set sample, where *y*_*i*_^*p*^ represents the *p*th image and the *i*-th medical image in the dataset, and *N* is the medical image total category. For medical image *Y* to be identified, the medical image classification system searches for an image of the same category by matching the medical image to be identified with the image category within the medical image system. Visual features and distance metrics are used to ensure that image pairs (*y*_*i*_, *y*_*i*_^+^) of the same medical category have a higher degree of similarity than image pairs (*y*_*i*_, *y*_*i*_^+^) of different medical categories. The original triple loss function is defined as follows [39, 40]:

(16) $$\begin{array}{c} L\left(y,w\right)=\overset{N}{\underset{i=1}{\sum }}\begin{array}{c} \max\left\{0,D\left(f\left(y_{i}\right),f\left(y_{i}^{+}\right)\right)\right.,\\ \left.-D\left(f\left(y_{i}\right),f\left(y_{i}^{-}\right)\right)+\alpha \right\}, \end{array} \end{array}$$

where D(.,.) is expressed as the Euclidean distance between two feature vectors. *α* represents the interval parameter. *w* represents a parameter in a deep convolutional network. The loss function will constrain the distance of the “dissimilar image pair” to be greater than the distance of the “similar image pair,” and the distance has a certain interval. However, when the feature distance of the image pair is very small, the gradient corresponding to each image will also become smaller. It may cause the disappearance of the back propagation time gradient, and it will learn a suboptimal model. In addition, the loss function does not restrict similar images to the distance within the class. It may make the features of the same medical category image have large clusters of intraclass variance in the learned feature space.

To solve the problem of the disappearance of the back propagation time gradient, the learning to obtain a suboptimal model and the loss function without constraints on the intraclass distance of similar image pairs. This paper proposes an improved triplet loss function to eliminate the defect that the original loss function has no adaptive ability. Its definition is as follows:

(17) $$\begin{array}{c} L\left(y,w,M\right)=\frac{1}{N}\overset{N}{\underset{i=1}{\sum }}\underset{\text{triplet}‐\text{wise constraint}}{\underbrace{\left(\max\left\{0,D_{x}\left(y_{i},y_{i}^{+},y_{i}^{-},w,M\right)\right\}\right)}}+\mu \cdot \underset{\begin{array}{cc} \text{pair}‐\text{wise} & \text{constraint} \end{array}}{\underbrace{D_{p}\left(y_{i},y_{i}^{+},y_{i}^{-},w,M\right)}}, \end{array}$$

where *N* represents the total number of input triplet images, *w* is a parameter in a deep convolutional network, *M* represents a Mahalanobis distance matrix, and *μ* represents a balanced weighting factor. The distance function *D*_*x*_, *D*_*p*_ is defined as follows:

(18) $$\begin{array}{c} D_{x}\left(y_{i},y_{i}^{+},y_{i}^{-},w,M\right)=\left(1-\frac{{\left\|f_{w}\left(y_{i}\right)-f_{w}\left(y_{i}^{-}\right)\right\|}_{M}^{2}}{{\left\|f_{w}\left(y_{i}\right)-f_{w}\left(y_{i}^{+}\right)\right\|}_{M}^{2}+\alpha }\right), \end{array}$$

(19) $$\begin{array}{c} D_{p}\left(y_{i},y_{i}^{+},w,M\right)={\left\|f_{w}\left(y_{i}\right)-f_{w}\left(y_{i}^{+}\right)\right\|}_{M}^{2}, \end{array}$$

where ‖·‖_*M*_^2^ represents the Mahalanobis distance between the two features. *α* represents the interval between predefined pairs of similar and dissimilar image pairs. The tripletwise constraint in the loss function belongs to the Mahalanobis distance of the matching pair whose Markov distance is less than the mismatched pair. Pairwise constraints are intended to constrain the distance between image features within a class, which makes the generated features robust to factors such as illumination, camera angle, blur, and occlusion. The improved triplet loss function is constrained in the distance between images, as shown in Figure 2. An improved triple loss function can be used to optimize the proposed deep convolutional neural network model. It can learn robust and discriminative medical image category feature information from the original image.

The proposed deep convolutional network model and the optimized triplet loss function are trained together by a stochastic gradient descent algorithm. The parameter *w* of the deep convolutional network model and the Mahalanobis distance matrix *M* are optimized. The learning process is iterated back and forth until the preset number of training rounds is reached, and an optimal network model is finally obtained. This optimization strategy is inspired by the optimization method [41]. This article replaces (*y*_*i*_, *y*_*i*_^+^, *y*_*i*_^−^) with *y*_*i*_ in the equation below. In each iteration, the Mahalanobis distance matrix *M* is first fixed as a constant, and the objective function becomes the optimized depth network model parameter *w*. Therefore, the optimized triplet loss function is simplified to optimize a similar form of the original triplet loss at the Euclidean distance. As network parameters are constantly updated and optimized, the network model can be extracted to obtain more efficient medical image feature representations. Formula (17) gives the calculation of the network parameter *w* partial derivative as follows:

(20) $$\begin{array}{c} \frac{\partial L\left(y,w,M\right)}{\partial w}=\frac{1}{N}\overset{N}{\underset{i=1}{\sum }}d_{x}\left(y_{i},w,M\right)+\frac{1}{N}\overset{N}{\underset{i=1}{\sum }}d_{p}\left(y_{i},w,M\right), \end{array}$$

(21) $$\begin{array}{c} d_{x}\left(y_{i},w,M\right)=\left\{\begin{array}{c} \frac{\partial D_{x}\left(y_{i},w,M\right)}{\partial w},D_{x}\left(y_{i},w,M\right)>0,\\ 0,D_{x}\left(y_{i},w,M\right)\leq 0, \end{array}\right. \end{array}$$

(22) $$\begin{array}{c} d_{p}\left(y_{i},w,M\right)=\mu \cdot \frac{\partial D_{p}\left(y_{i},w,M\right)}{\partial w}. \end{array}$$

According to *D*_*x*_(*y*_*i*_, *w*, *M*) and *D*_*p*_(*y*_*i*_, *w*, *M*) defined in the previous formula, their gradient formulas for *w* are as follows:

(23) $$\begin{array}{c} \frac{\partial D_{x}\left(y_{i},w,M\right)}{\partial w}=\tilde{M}\left(f_{w}\left(y_{i}\right)-f_{w}\left(y_{i}^{-}\right)\right)\frac{\partial f_{w}\left(y_{i}\right)-\partial f_{w}\left(y_{i}^{-}\right)}{\partial w}g_{1}+\tilde{M}\left(f_{w}\left(y_{i}\right)-f_{w}\left(y_{i}^{+}\right)\right)\frac{\partial f_{w}\left(y_{i}\right)-\partial f_{w}\left(y_{i}^{+}\right)}{\partial w}g_{2}, \end{array}$$

(24) $$\begin{array}{c} \frac{\partial D_{p}\left(y_{i},w,M\right)}{\partial w}=\tilde{M}\left(f_{w}\left(y_{i}\right)-f_{w}\left(y_{i}^{+}\right)\right),\frac{\partial f_{w}\left(y_{i}\right)-\partial f_{w}\left(y_{i}^{+}\right)}{\partial w}, \end{array}$$

where $\tilde{M}=\left(M+M^{T}\right)$, *g*_1_ = −(‖*f*_*w*_(*y*_*i*_) − *f*_*w*_(*y*_*i*_^−^)‖_*M*_^2^ + *α*)/(‖*f*_*w*_(*y*_*i*_) − *f*_*w*_(*y*_*i*_^+^)‖_*M*_^2^ + *α*)^2^, *g*_2_ = (‖*f*_*w*_(*y*_*i*_) − *f*_*w*_(*y*_*i*_^−^)‖_*M*_^2^ + *α*)/(‖*f*_*w*_(*y*_*i*_) − *f*_*w*_(*y*_*i*_^+^)‖_*M*_^2^ + *α*)^2^. It can be seen from equations (23) and (24) that in the case of given eigenvalues *f*_*w*_(*y*_*i*_), *f*_*w*_(*y*_*i*_^+^), and *f*_*w*_(*y*_*i*_^−^) and gradients *∂f*(*y*_*i*_)/*∂w*, *∂f*(*y*_*i*_^+^)/*∂w*, and *∂f*(*y*_*i*_^−^)/*∂w*, the gradient of each image in the triple is calculated. Therefore, the Mahalanobis distance matrix *M* is fixed to a constant. The gradient update for *w* in formula (17) can be obtained by standard forward and backward propagation through the network model for each image in the triple.

After this phase of each round of iterations, all training images can be mapped to a particular feature space by training the updated deep network model. In the second stage, given a triplet image feature representation *f*_*w*_(*y*_*i*_), *f*_*w*_(*y*_*i*_^+^), and *f*_*w*_(*y*_*i*_^−^), the objective function becomes a semipositive distance measure matrix *M* optimized in formula (17), which is used to map feature representations from feature spaces to appropriate distance spaces. Therefore, it can use an iterative gradient random descent projection algorithm to optimize the objective function. Specifically, at each iteration, the parameter *M* is optimized along the direction of the gradient descent to reduce the target loss. The matrix *M* is then projected onto a feasible set containing all of its semipositive definite matrices *S*_+_. The formula for calculating the partial derivative of the Mahalanobis distance matrix *M* in formula (17) is as follows:

(25) $$\begin{array}{c} \frac{\partial L\left(y,w,M\right)}{\partial M}=\frac{1}{N}\overset{N}{\underset{i=1}{\sum }}d_{x}^{*}\left(y_{i},w,M\right)+\frac{1}{N}\overset{N}{\underset{i=1}{\sum }}d_{p}^{*}\left(y_{i},w,M\right), \end{array}$$

(26) $$\begin{array}{c} d_{x}^{*}\left(y_{i},w,M\right)=\left\{\begin{array}{c} \frac{\partial D_{x}\left(y_{i},w,M\right)}{\partial M},D_{x}\left(y_{i},w,M\right)>0,\\ 0,D_{x}\left(y_{i},w,M\right)\leq 0, \end{array}\right. \end{array}$$

(27) $$\begin{array}{c} d_{p}^{*}\left(y_{i},w,M\right)=\mu \cdot \frac{\partial D_{p}\left(y_{i},w,M\right)}{\partial M}. \end{array}$$

Given the *D*_*x*_(*y*_*i*_, *w*, *M*) and *D*_*p*_(*y*_*i*_, *w*, *M*) conditions, their gradient formulas for parameter matrix *M* are as follows:

(28) $$\begin{array}{c} \frac{\partial D_{x}\left(y_{i},w,M\right)}{\partial M}=g_{1}\cdot C_{{ii}^{-}}+g_{2}\cdot C_{{ii}^{+}}, \end{array}$$

(29) $$\begin{array}{c} \frac{\partial D_{p}\left(y_{i},w,M\right)}{\partial M}=C_{{ii}^{+}}, \end{array}$$

where *C*_*ij*_ = (*f*(*y*_*i*_) − *f*(*y*_*j*_)) (*f*(*y*_*i*_) − *f*(*y*_*j*_))^*T*^. Minimizing formula (17) in the process of optimizing *M*, it must ensure that matrix *M* is a semipositive definite matrix. Thus, the gradient updated matrix *M* is projected onto cone *S*_+_, which includes all semidefinite matrices after each gradient iteration. The projection process is achieved by matrix diagonalization. The formula *M* = *V*Δ*V*^*T*^ represents an eigenvalue decomposition operation on the distance metric matrix *M*. *V* represents an orthogonal matrix of eigenvectors of the metric matrix. ∆*b* denotes a diagonal matrix of the composition of the eigenvalues of the metric matrix. The diagonal matrix can be further split into Δ = Δ^+^ + Δ^−^. Δ+ contains all positive eigenvalues; Δ− contains all negative eigenvalues. Matrix *M* is then projected onto the cone in mathematical form as:

(30) $$\begin{array}{c} P_{S_{+}}=V\Delta^{+}V^{T}. \end{array}$$

Formula (29) rejects all negative eigenvalues of matrix *M* after each iteration update by zeroing the negative eigenvalues. It guarantees the semidefiniteness of the matrix *M*.

The optimization algorithm of formula (17) optimizes the depth network model parameter *w* and the Mahalanobis distance matrix *M* using the update rules in formulas (20), (25), and (29). The main learning process: first, from the initialization of *M* and *w*, set *M* as the unit matrix and train according to the predefined number of iterations. In the first stage, the Mahalanobis distance matrix *W* in formula (17) is first fixed, and then the network parameter *w* is optimized using a small batch gradient random descent algorithm. In the second phase, the parameter *w* is fixed, and the medical classification image is transferred to the feature space through the updated depth network model. Then, the iterative Mahalanobis distance matrix *M* is optimized using formulas (25) and (29) in the gradient projection algorithm. After multiple rounds of iterative optimization, the optimized deep convolutional neural network model and the appropriate metric matrix *M* are obtained at the same time.

### 3.4. Triad Sampling

Assuming that the dataset has *N* medical image categories and that each medical category image has *M* images, the number of all possible triples will reach *N*(*N* − 1)*M*^2^(*M* − 1). It is impractical to load a large number of triples into the computer's memory at once. Therefore, a valid triple sampling strategy must be selected in the model to generate the appropriate number of triples, and a batch triple sampling strategy is used to optimize the training network model. This paper presents an effective triad sampling strategy. For each batch input, this paper randomly extracts *K* categories, and each category randomly samples *L* images to form a batch input. Therefore, the batch input contains *K*∙*L* images. For each image sample in the batch input, we select the most difficult positive sample (the same category image with large intraclass differences) and the most difficult negative samples (images that look similar but of different categories) from a triple. The number of triples generated in this way is moderate, as only the most difficult samples in the batch input are selected, which reduces training time and ensures that the network can learn to express feature representations with resolution. At each iteration, a fixed number of batch inputs are sent to the network model. As the number of iterations increases, the network model covers all samples and converges to optimal values.

## 4. Medical Classification Algorithm Based on a Visual Attention Mechanism-Multiscale Convolutional Neural Network

Based on the above, this section builds a medical classification algorithm based on the visual attention mechanism-multiscale convolutional neural network. First, the visual attention mechanism is introduced to fully exploit the characteristics of medical images. It solves the effective positioning and extraction of medical image feature information and increases the interpretable type of model. Then, this paper constructs a novel multiscale convolutional neural network model that can automatically extract high-level discriminative appearance features from the original image so that network learning can obtain more effective medical image feature information. It can improve the robust performance of the network model. Finally, a medical classification algorithm based on a visual attention mechanism-multiscale convolutional neural network is established. The algorithm is used to complete the medical image classification task. The basic flowchart of the proposed medical image classification algorithm is shown in Figure 3. The basic steps are as follows:

1. First, the medical image data are subjected to preprocessing, such as denoising
2. The deep learning model based on a visual attention mechanism is used to visualize attention and increase the interpretable model. It can solve the relevance problem. Compared with other methods, it solves the effective positioning and extraction of medical image feature information
3. To solve the problem of matching the deep learning network structure and training strategy to medical images, this paper constructs a novel multiscale convolutional neural network model. It can automatically extract high-level discriminative appearance features from the original image, and the loss function uses the Mahalanobis distance optimization model to obtain a better training strategy. It improves the robust performance of the network model
4. The method in step (2) to step (3) is introduced. A medical classification algorithm based on a visual attention mechanism-multiscale convolutional neural network is established through steps (1)–(3). The medical image classification algorithm is used to analyze related examples to obtain classification results

## 5. Example Analysis

### 5.1. Lung Nodule Classification Experiment

To verify the effect of the proposed algorithm on medical image classification, this section classifies and tests the lung nodule database established by the Japanese Society of Radiology Technology (JSRT) [42]. This algorithm is compared with other mainstream medical image classification algorithms.

#### 5.1.1. Database Introduction and Test Process Description

The lung nodule database established by JSRT was confirmed by CT imaging, and the location information of lung nodules was confirmed by three chest radiologists. The lung nodule database established by JSRT has a total of 247 chest radiographs from 15 different medical institutions in the world, including 154 cases of pulmonary nodules and 93 cases of no pulmonary nodules. The size of each image in the database is 2048 × 2048 pixels. The diameter of the lung nodules ranges from 5 to 40 mm. The lung nodule database established by JSRT is classified as very obvious, obvious, inconspicuous, not obvious, and extremely inconspicuous according to the degree of detection of pulmonary nodules. In this experiment, only the lung nodules in the obvious area of the lung were classified. A total of 150 lung nodule images met the test criteria. Some example pictures are shown in Figure 4.

To better serve the later classification test, for the lung nodule database established by JSRT, this experiment used the gray histogram method to enhance the experimental image, as shown in Figure 5. The enhanced image can greatly improve the contrast of the lung nodules and the surrounding tissue structure.

The deep learning model used in this experiment was based on the PyTorch implementation and was trained on a Titan-X GPU. The deep learning model was based on the visual attention mechanism-multiscale convolutional neural network proposed in Sections 2 and 3 of this paper. The initial learning rate was set to 0.01, the learning rate was reduced to one-tenth of the original when training was conducted to 50 and 80 epochs, and the training lasted for 160 epochs. In all training sessions, the model proposed in this paper was trained based on the stochastic gradient descent method, and the number of samples per batch was set to 128.

#### 5.1.2. Classification Results and Analysis

The medical image classification algorithm proposed in this paper and other mainstream medical image classification algorithms were used to classify the lung nodule database established by JSRT. The classification results are shown in Table 1.

Table 1 shows that the classification accuracy of the medical classification algorithm based on the visual attention mechanism-multiscale convolutional neural network proposed in this paper improved compared with the traditional machine learning algorithm and other deep learning algorithms. This method has certain advantages. Specifically, the traditional machine learning methods proposed in [43, 44] have classification accuracy rates of 95.37% and 95.96%, respectively. Although the classification accuracy of traditional machine learning methods reached 95%, traditional machine learning methods are still the least effective among the listed classification methods because the traditional machine learning method has certain problems in the training effect of the lung nodule database established by JSRT, which directly leads to the image classification accuracy being weaker than other categories. The recognition accuracy of the deep learning method proposed in the literature [45–47] was 98.12%, 98.23%, and 98.38%, respectively. Their classification accuracy was above 98%, and the classification accuracy was higher than the traditional machine learning method by more than 1%. This is mainly because the deep learning model can train the lung nodule database established by JSRT to obtain a more reasonable and reliable image classification model. The classification accuracy of this method was 99.86%, and the classification accuracy rate was the highest among all methods, which is close to all accurate classifications, which fully verifies that the proposed method can improve the accuracy of image classification and has better stability and robustness. This is mainly because the method proposed in this paper compared the method proposed in [43–47], and not only introduced the visual aid mechanism to the deep learning model but also improved the network structure and loss function in the deep learning model. Through the optimization and improvement of the two, the modeling ability and nonlinear classification ability of the deep learning model improved, and the highest classification effect was achieved.

### 5.2. Breast Cancer Classification Experiment

To further verify the effect of the proposed algorithm on medical image classification, this section classifies and tests the Wisconsin Breast Cancer Database (WBCD) [48] and compares it with mainstream medical image classification algorithms.

#### 5.2.1. Database Introduction and Test Process Description

The WBCD was established by the University of California, Irvine, and the WBCD has a total of 699 human breast tissue samples. Of these, 458 samples were benign, and 241 samples were malignant. All samples consisted of 9 cytological features of benign or malignant breast fine-needle aspiration. Each feature determines a specific value based on how well the sample is expressed on the feature, and values are integer values between 1 and 10. Additionally, since the dataset includes 16 samples lacking specific attribute values, considering the lack of samples with missing data values, they are treated as invalid data in the experiments in this paper. Only relevant experiments were performed on the remaining 683 samples.

The deep learning model used in this experiment was based on the PyTorch implementation and was trained on the Titan-X GPU. The deep learning model is based on the visual attention mechanism-multiscale convolutional neural network proposed in Sections 2 and 3 of this paper. The initial learning rate was set to 0.001, and the batch size was 16. The momentum was set to 0.3, and the weight attenuation parameter was set to 0.0004. All dimensions were set for each pooled size, and stride was set to 2.

#### 5.2.2. Classification Results and Analysis

The WBCD database was classified and identified by the medical image classification algorithm proposed in this paper and other mainstream medical image classification algorithms. For a more fair comparison, this experiment used the average accuracy of the training test ratio of 1 : 1 and the training test ratio of 2 : 1. Each was the result of 20 averages. The classification results are shown in Table 2.

Table 2 shows that the classification accuracy of the medical classification algorithm based on the visual attention mechanism-multiscale convolutional neural network proposed in this paper improved compared with the traditional machine learning algorithm and other deep learning algorithms. This method has obvious advantages. Specifically, the traditional machine learning methods proposed in [49–51] had classification accuracy rates of 92.78%, 93.39%, and 95.61%, respectively. Although the classification accuracy of traditional machine learning methods reached more than 92%, the traditional machine learning method still had the lowest recognition accuracy among the listed classification methods because the traditional machine learning method has a poor training effect on the WBCD database. The recognition accuracy of the deep learning method proposed in the literature [52–54] reached 98.53%, 99.02%, and 99.23%, respectively. Their classification accuracy rate was over 98%, which was more than 3% higher than traditional machine learning methods because the deep learning model obtained a more reasonable and reliable image classification model for WBCD database training. The classification accuracy of this method was 99.89%, and the classification accuracy rate was the highest among all methods, which was similar to all accurate classifications. It fully verifies that the proposed method can extract the various feature information of the WBCD database to the maximum extent. It further proves that the deep learning model proposed in this paper is better than the deep learning method proposed in [52–54]. This is mainly because the proposed method can better optimize the network architecture of the deep learning model and introduce the visual attention mechanism.

In summary, experiments using lung nodules and breast cancer medical image databases show that the traditional medical image classification algorithm has the disadvantages of low recognition accuracy and poor stability in medical image classification tasks. The classification accuracy of the deep learning classification algorithm in the above database is significantly better than that of the traditional machine learning algorithm. This proves the advantages of the deep learning model. In addition, the medical image classification algorithm based on the visual attention mechanism-multiscale convolutional neural network proposed in this paper can obtain better classification performance than other proposed deep classification algorithms because the deep learning model proposed in this paper not only solves the problem of model network architecture but also introduces a visual attention mechanism that is particularly effective for medical image classification.

## 6. Conclusion

Since medical images have more distinct and different feature information than natural images, medical image characteristics must be fully considered in establishing a deep learning model for medical image classification. Therefore, this paper first adds the visual attention mechanism to the deep learning model, and the attention mechanism increases the explanatory form of the model by visualizing the attention, which can extract the feature information of the medical image more effectively. To solve the problem of matching the deep learning network structure and training strategy to medical images, a novel multiscale convolutional neural network model is constructed. It automatically extracts high-level discriminative appearance features from the original image and improves the robust performance of the network model. Based on this, this paper proposes a medical classification algorithm based on a visual attention mechanism-multiscale convolutional neural network.

The results of lung nodule and breast cancer classification experiments show that the classification accuracy of the deep learning medical image classification method is the highest, reaching 99.86% and 99.89%. This is because this paper better solves the problem of the network structure of the deep learning model and the interpretability of the model. Additionally, the deep learning medical image classification method proposed in this paper can extract the feature information of medical images better, which is beneficial for improving the effects of lung nodules and breast cancer classification experiments. Therefore, the deep learning medical image classification method proposed in this paper achieves the best classification accuracy.

## Figures and Tables

**Figure 1:** The overall framework of multiscale CNN.

**Figure 2:** Schematic diagram of the optimized triplet loss function versus image distance constraint.

**Figure 3:** Basic flowchart of the medical classification algorithm based on a visual attention mechanism-multiscale convolutional neural network.

**Figure 4:** Part of the lung nodule image.

**Figure 5:** Comparison of lung nodules before and after image enhancement.

**Table 1:** Comparison table of classification results of different classification algorithms on the lung nodule database established by JSRT (%).

Method type	Classification accuracy
[43]	95.37
[44]	95.96
[45]	98.12
[46]	98.23
[47]	98.38
Our	99.86

**Table 2:** Comparison table of classification results of different classification algorithms on the WBCD database (%).

Method type	Classification accuracy
Rough cotraining [49]	92.78
Bayesian [50]	93.39
Neural networks [51]	95.61
CNN [52]	98.53
DeepNet1 [53]	99.02
DeepNet2 [54]	99.23
Our	99.89

## Data Availability

The data used to support the findings of this study are included within the paper.
